# Comparison of Dizziness Factors for Mild Traumatic Brain Injury Patients with and without Dizziness: A Factor Analysis and Propensity Score Model Study

**DOI:** 10.1155/2021/5571319

**Published:** 2021-05-11

**Authors:** Hon-Ping Ma, Jiann Ruey Ong, Ju-Chi Ou, Yung-Hsiao Chiang, Shoou-Yang Lian

**Affiliations:** ^1^Emergency Department, Shuang Ho Hospital, Taipei Medical University, Taiwan; ^2^Emergency Department, School of Medicine, Taipei Medical University, Taiwan; ^3^Graduate Institute of Injury Prevention and Control, Taipei Medical University, Taiwan; ^4^Department of Surgery, College of Medicine, Taipei Medical University, Taipei, Taiwan; ^5^Department of Neurosurgery, Taipei Medical University Hospital, Taipei, Taiwan; ^6^Neuroscience Research Center, Taipei Medical University, Taipei, Taiwan; ^7^Department of Emergency, Yuan's General Hospital, Taiwan

## Abstract

Traumatic brain injury (TBI) causes major socioeconomic problems worldwide. In the United States, nearly three-quarters of patients with TBI have mild TBI (mTBI). 32% of these patients may develop dizziness. In this study, we analyzed the factor structure of the traditional Chinese version of the DHI and evaluate the differences in DHI factors between dizziness and nondizziness groups. In total, 315 patients with mTBI, comprising 158 with self-reported dizziness and 157 without dizziness, were recruited from three hospitals. The responses for Beck Depression Inventory (BDI), Beck Anxiety Inventory (BAI), Epworth Sleepiness Scale (ESS), and Pittsburgh Sleep Quality Index (PSQI) demonstrated between-group differences. The Chinese DHI had internal validity and had four factors that differed from the English version (3 aspects). The group effects for the physical subscale remained significantly different even after adjustments in the propensity score model. For the Chinese version, two of four factors remained significantly different in the effects between self-reported dizziness and nondizziness groups. The factors of our Chinese DHI differed from those of the original English version of DHI. After adjustments using the propensity score model, the physical subscale demonstrated significant differences between the self-reported dizziness and nondizziness groups. Only two factors from our Chinese DHI were significantly different; moreover, it contained only three physical, five functional, and three emotional items.

## 1. Introduction

Traumatic brain injury (TBI) is a leading cause of death and disability. Of all 25-year-old patients with TBI, 33% require medical attention [1, 2]. TBI symptoms are typically assessed on the Glasgow Coma Scale (GCS), which classifies TBI as mild, moderate, or severe. In the United States, nearly three-quarters of patients with TBI have mild TBI (mTBI) [3]. The common causes of mTBIs are vehicle accidents, accidents or injuries during military deployment, athletic activities, and falls [4]. A person with an mTBI may experience headaches, dizziness, sleep disorders, mood changes, or lose consciousness for a few minutes [5]. Thirty-two percent of patients experience dizziness for >2 weeks after injury, in addition to anxiety, depression, or poor sleep quality [6, 7]. Of these, dizziness has been reported as a contributor to both short- and long-term disability after an mTBI [8].

The Dizziness Handicap Inventory (DHI), commonly used to evaluate balance impairment and disability level in a nonspecific patient population [9], contains 25 self-reported items used to score dizziness based on three domains: physical (0–28 points), emotional (0–36 points), and functional (0–36 points). The DHI, originally in English, has been translated into Dutch, Spanish, and Japanese [10–15].

In this study, the factor structure of the DHI was investigated using data from a sample of patients with mTBI. Factor analysis was used to determine the internal consistency and reliability of our traditional Chinese version of the DHI (hereafter, our Chinese DHI) and confirm the validity of its content domains. Furthermore, the differences in our Chinese DHI domains between self-reported dizziness and nondizziness groups were evaluated using a propensity score model.

## 2. Methods

### 2.1. Participants

Patients with mTBI aged 20–70 years who visited the emergency departments of Taipei Medical University Hospital, Taipei Municipal Wanfang Hospital (managed by Taipei Medical University), or Taipei Medical University Shuang Ho Hospital from May 2010 to May 2014, were recruited. Only the patients proficient in the Chinese language and with GCS scores of 13–15, no remarkable computed tomography imaging findings, and loss of consciousness for <30 minutes were included. The exclusion criteria were pregnancy and past history of TBI and mental illness. Patients who met the inclusion criteria were referred to study nurses by the physicians at the aforementioned emergency departments with two weeks postbrain injury. Taipei Medical University–Joint Institutional Review Board approved the study protocol (No.201003008). In total, 315 patients with mTBI agreed to join this study, signed the informed consent form, and completed this study without missing. The self-reported dizziness defined as a patient answer “yes” for the following question: have you felt dizziness since mild traumatic brain injury?

### 2.2. Measures

The DHI is a validated 25-item questionnaire that grades the extent to which dizziness affects daily life [16]. This original English version has three domains: functional (0–36 points), emotional (0–36 points), and physical (0–28 points). Each domain has questions with three possible responses: “no,” “sometimes,” and “yes,” which are scored as 0, 2, and 4, respectively. The total score of DHI also was calculated by summarizing all three domains, and a higher score indicated more serious problems. The Chinese version of DHI was found to have good test–retest reliability and internal consistency—comparable to those of the original DHI [17].

Four questionnaires were collected as confounders, including Beck Anxiety Inventory (BAI), Beck Depression Inventory (BDI), Epworth Sleepiness Scale (ESS), and Pittsburgh Sleep quality index (PSQI). The Beck Anxiety Inventory (BAI) and Beck Depression Inventory (BDI), developed by Aaron T. Beck, are self-administered questionnaires consisting of 21 multiple choice questions that measure the magnitude of anxiety and depression symptoms [18, 19]. For each question, the scores range from 0 (not at all) to 3 (severe), and the total score ranges from 0 to 63. The Epworth Sleepiness Scale (ESS) is a self-administered questionnaire, comprising eight questions that survey the likelihood of daytime sleepiness [20]. Each question is a score from 0 (would never doze) to 1 (slight chance of dozing), 2 (moderate chance of dozing), and 3 (high chance of dozing). The total score ranges from 0 to 24, with a score of 11-24 indicating excessive daytime sleepiness. The Pittsburgh Sleep Quality Index (PSQI), which measures the quality and patterns of sleep over the course of a month, contains 19 questions related to seven components including, namely, subjective sleep quality, sleep latency, sleep duration, habitual sleep efficiency, sleep disturbance, use of hypnotics, and daytime dysfunction [21]. PSQI scores range from 0 (no problem) to 3 (serious problem), with a maximum global PSQI score of 21 points indicating severe sleep dysfunction. The higher score indicated a more serious problem for all four questionnaires, and the Chinese version of the BAI, BDI, ESS, and PSIQ was validated, respectively [22–25].

### 2.3. Statistical Analysis

The baseline characteristics of patients with and without dizziness were compared using the Mann–Whitney *U* test, a nonparametric test, for continuous variables and the *χ*^2^ test for categorical variables. The internal consistency of our Chinese DHI was evaluated using Cronbach's *α* and corrected item-total correlations (CI-TCs). Kaiser–Meyer–Olkin (KMO) and Bartlett's tests were used to evaluate variables for factor analysis. The dimensions of our Chinese DHI were evaluated using principal component analysis (PCA) with orthogonal rotation. Factors with eigenvalues >1 (i.e., Kaiser's criterion) were extracted, and the cutoff point corresponded to the inflection point of the curve in the scree plot. At least four-factor loadings were >0.6, and four questions were a minimum requirement for each factor [26, 27]. The correlations were assessed using the Pearson correlation coefficient, resulting in values between +1 and −1. The propensity score model was used to address the effect of potential confounding variables in an observational study with the goal of reducing bias in the estimates [28]. The propensity score is primarily applied to matching, stratification, and weighting and as a variable [29, 30]. The difference of new dimensions of our Chinese DHI between self-reported dizziness and nondizziness group was evaluated using a propensity score model. All analyses were performed using R. A *P* value of <0.05 was considered statistically significant.

## 3. Results

### 3.1. Characteristics of the Patients

We included 315 patients with mTBI, 158 (50.16%) of whom had self-reported dizziness (Table 1). No differences were noted between the self-reported dizziness and nondizziness groups in the following variables: age, education year, smoker, drinker, and GCS. However, the proportion of male patients was significantly lower in the self-reported dizziness group (46.29%) than in the nondizziness group (77.49%); similarly, the proportion of patients with headaches was significantly higher in the self-reported dizziness group (77.22%) than that in the nondizziness group (34.39%).

### 3.2. Questionnaires Results

The scores of the self-reported dizziness and nondizziness groups for all included confounders demonstrated significant differences (Table 2). The average scores for all questionnaires were higher in the self-reported dizziness group than in the nondizziness group. The average BAI, BDI, ESS, and PSQI were 12.59, 11.25, 7.99, and 8.49 in the self-reported dizziness group and 4.81, 6.39, 6.39, and 4.36, in the nondizziness group. On the other hand, the measurement of dizziness, DHI, showed a significant difference in the total score of DHI between self-reported dizziness and self-reported nondizziness groups. The differences of all three domains between dizziness and nondizziness groups were statistically significant. For the emotional domain of original DHI, the average scores were 11.27 (±8.19) and 5.86 (±7.56) for dizziness and nondizziness groups, respectively. For the functional domain of original DHI, the average scores were 14.22 (±9.65) and 8.08 (±10.08) for dizziness and nondizziness groups. For the physical domain of original DHI, the average scores were 12.36 (±7.09) and 6.29 (±6.65) for dizziness and nondizziness groups.

### 3.3. Factor Analysis

#### 3.3.1. Internal Consistency

Table 3 presents the means scores (standard deviations) and CI-TC coefficients for all DHI items. The strength of the relationship between a single item and all remaining items was measured using CI-TCs. The CI-TC coefficients ranged from 0.42 (item 15: afraid people think you are intoxicated) to 0.74 (item 6: restrict participation in social activities) for the total DHI score, from 0.62 (item 4: walk down supermarket aisle) to 0.73 (item 25: bend over) for the DHI-physical subscore, from 0.52 (item 15: afraid people think you are intoxicated) to 0.71 (item 9: afraid to leave home alone) for the DHI-emotional subscore, and from 0.59 (item 12: avoid heights) to 0.80 (item 6: restrict participation in social activities) for the DHI-functional subscore. The KMO value was 0.94, and *P* for Bartlett's test was <0.001, confirming that the factor analysis was appropriate for the set of variables in this study. The two-, three-, four-, and five-factor solutions accounted for 45%, 48%, 51%, and 54% of the variance, respectively.

The graphical representation of the eigenvalues is shown in Figure 1. According to the scree plot, a four-factor model was selected. The list of new factors (T1, T2, T3, and T4) and the corresponding factor loading are presented in Table 4.

The first factor (T1) consisted of four physical items, two functional items, and two emotional items. The first factor had five items with a factor loading of >0.6: quick head movement, bend over, job or household responsibilities, hard to concentrate, and depressed. The second factor (T2) comprised nine items with two functional items, one physical item, and six emotional items. The T2 had two items with a factor loading of >0.6: afraid to stay home alone and stressed relationship with family/friends.

The third factor (T3) and the fourth factor (T4) consisted of five and four items, respectively. The T3 included two functional items and three physical items, and none of the T3 items has a factor loading of >0.6. The T4 factor included one emotional item and three functional items—and the item Restrict travel with a factor loading of >0.6.

### 3.4. Difference Evaluation via a Propensity Score Model

The correlation coefficients for all questionnaires are listed in Table 5. All four questionnaires, BAI, BDI, ESS, and PSQI, were significantly correlated with the total DHI and its subscales as well as with both the Japanese and Chinese versions of DHI. The two patient groups were imbalance in BAI, BDI, ESS, and PSQI. Therefore, the propensity score model included age, sex, BAI, BDI, ESS, and PSQI. The group effect was evaluated both with and without the propensity scores. The results of regression analysis of the models with and without propensity scores are presented in Table 6. A total of eight outcomes were evaluated: total DHI, DHI-functional, DHI-physical, DHI-emotional, T1, T2, T3, and T4. The group effects were significant for all eight outcomes before propensity score adjustments. All eight scores of the self-reported dizziness group were higher (i.e., positive group effects) than those of the nondizziness group. After propensity score adjustments, four of the eight outcomes differed significantly between the groups: DHI-total score, DHI-physical, T1, and T4. T1 consisted of three items in the physical domain (“Perform more ambitious activities”, “Quick head movements”, “Bend over”), two items in the functional domain (“strenuous homework or yard work”, “Job or household responsibilities”), and two items in the emotional domain (“Hard to concentrate”, “Depressed”). T4 included one item in the emotional domain (“Feel frustrated”) and three items in the functional domain (“Restrict travel”, “Restrict participation in social activities”, “Hard to read”).

## 4. Discussion

Four factors of our Chinese DHI were a suggestion from our dataset. The factor analyses of the original, Dutch, Spanish, German, and Japanese versions of the DHI thus far have provided more than one-factor solutions [10–12, 14]. The original DHI was designed with three subscales: physical, functional, and emotional. For distinct study-population and sample-size compositions, the factors of our Chinese DHI differ from those of the original and Japanese versions. T1 included three items in the J2 (Japanese factor 2) and J3 (Japanese factor 3) and one in the J1 (Japanese factor 1). T2 consisted of four items in J1, three items in J4 (Japanese factor 4), and two items in J2. T3 included two items in J1, two in J5 (Japanese factor 5), and one in J3. T4 factor included with three items in J1 and one in J2. Moreover, sample populations used to verify the DHI have varied in their dizziness etiologies: for verification of the original DHI version, individuals with Meniere's disease were included [10], whereas for the verification of the Japanese version, patients with bilateral peripheral vestibular dysfunction, central vestibular dysfunction, or unilateral peripheral vestibular dysfunction were included [15]. By contrast, here, we included patients with first-time mTBIs and self-reported dizziness.

In summary, the significant factors of our Chinese DHI for patients with mTBIs were different than that of the original DHI. Two of the four factors showed significant differences between the self-reported dizziness and nondizziness groups—with one factor including “Perform more ambitious activities,” “Quick head movements,” “Bend over,” “Strenuous housework or yard work,” “Job or household responsibilities,” “Hard to concentrate,” and “Depressed” and the other including “Feel frustrated,” “Restrict travel,” “Restrict participation in social activities,” and “Hard to read.”

The factor analysis for dizziness is relevant to prevent dementia. Several cohort studies have reported the absence of a relationship between self-reported mTBI and dementia risk [31, 32]. Nevertheless, a cohort study indicated that TBI severity and dementia diagnosis are associated and that mTBI without loss of consciousness increases dementia risk [33]. This was corroborated by another study, where patients with dizziness demonstrated a high dementia risk [34]. The major symptoms of patients with mTBI include depression, sleep disturbance, headache, dizziness, and anxiety [35–37]. A quasiexperiment was conducted using the propensity score model to assess the group effects in the current study. After the underlying confounding variables were balanced, the physical subscale became significantly different between our dizziness and nondizziness groups. Only two factors of our Chinese DHI demonstrated significant differences between the dizziness and nondizziness groups: the first significant factor included three physical, two functional, and two emotional items, whereas the second significant factor included one emotional and three functional items.

Dizziness, one of the neurosensory symptoms, was found in the elderly frequently and even more in elderly patients with dementia for prevalence varying from 14.2% to 77.5% [38–42]. The neurobehavior consequences, such as psychiatric and neurodegenerative disease of mTBI patients, may be persisted [43–46]. Therefore, the understanding of dizziness structure might be important for rehabilitation in advance for the aging society.

This study has some limitations. First, our patients with mTBI were all recruited from the emergency department, none of whom were existing inpatients or outpatients. Therefore, the current patient population may not represent all patients with mTBIs. Second, dizziness was self-reported, which may have led to reporting bias. Future studies investigating the constructs of the Chinese DHI further after considering the present limitations are warranted. In addition, factors such as vertigo, dizziness, and imbalance may be considered when recruiting patients.

## 5. Conclusion

The factors of our Chinese DHI differed from those of the original English version of DHI. The physical subscale in the English version demonstrated significant differences between the self-reported dizziness and nondizziness groups. Two factors from the Chinese DHI, containing three physical, five functional, and three emotional items were significantly different between the two groups.

## Figures and Tables

**Figure 1:** Scree plot of eigenvalues.

**Table 1:** Characteristics of the study population (mean standard deviation).

	mTBI	Dizziness	Nondizziness	*P* value
Sample size (*n*)	315	158	157	
Age	39.62 ± 14.45	39.00 ± 14.23	40.23 ± 14.70	0.50
Male (*n*, %)	123,39.05%	46,29.11%	77,49.04%	<0.01
Education (year)	13.21 ± 3.11	13.31 ± 3.35	13.12 ± 2.86	0.26
Headache (*n*, %)	176,55.87%	122,77.22%	54,34.39%	<0.01
Smoke (*n*, %)	95,30.16%	44,27.85%	51,32.48%	0.25
Drink (*n*, %)	144,45.71%	67,42.41%	77,49.04%	0.11
GCS	14.97 ± 0.34	14.99 ± 0.11	14.94 ± 0.47	0.65

GCS: Glasgow Coma Scale.

**Table 2:** Results of questionnaires of the study population (mean standard deviation).

	mTBI	Dizziness	Nondizziness	*P* value
BAI	8.69 ± 9.28	12.59 ± 10.82	4.81 ± 5.06	<0.01
BDI	8.81 ± 8.19	11.25 ± 8.70	6.39 ± 6.87	<0.01
ESS	7.46 ± 4.36	7.99 ± 4.58	6.93 ± 4.09	0.04
PSQI	7.58 ± 4.07	8.49 ± 6.68	4.36 ± 3.55	<0.01
DHI-total	29.01 ± 24.17	37.85 ± 22.59	20.23 ± 22.48	<0.01
DHI-emotional	8.56 ± 8.32	11.27 ± 8.19	5.86 ± 7.56	<0.01
DHI-functional	11.14 ± 10.32	14.22 ± 9.65	8.08 ± 10.08	<0.01
DHI-physical	9.31 ± 7.50	12.36 ± 7.09	6.29 ± 6.65	<0.01

BAI: Beck's Anxiety Inventory; BDI: Beck's Depression Inventory; ESS: Epworth Sleepiness scale; PSQI: Pittsburgh Sleep Quality Index; DHI: Dizziness Handicap Inventory.

**Table 3:** Means and standard deviation (SD) of items and corrected item-total correlation.

DHI		Abbreviation	Mean	SD	CI-TC			
					Total	Physical	Emotional	Functional
1	P	Look up	1.14	1.4	0.57	0.63		
2	E	Feel frustrated	1.83	1.6	0.73		0.64	
3	F	Restrict travel	1.74	1.7	0.71			0.74
4	P	Walk down supermarket aisle	0.72	1.3	0.65	0.62		
5	F	Get into or out of bed	1.03	1.5	0.65			0.65
6	F	Restrict participation in social activities	1.32	1.7	0.74			0.80
7	F	Hard to read	1.46	1.6	0.63			0.66
8	P	Perform more ambitious activities	1.61	1.6	0.64	0.68		
9	E	Afraid to leave home alone	1.04	1.6	0.70		0.71	
10	E	Embarrassed in front of other	0.55	1.2	0.51		0.49	
11	P	Quick head movements	2.43	1.7	0.62	0.67		
12	F	Avoid heights	1.34	1.7	0.62			0.59
13	P	Turning over in bed	0.92	1.5	0.56	0.58		
14	F	Strenuous homework or yard work	1.38	1.7	0.71			0.75
15	E	Afraid people think you are intoxicated	0.58	1.3	0.42		0.52	
16	F	Go for a walk by yourself	0.69	1.3	0.60			0.61
17	P	Walk down a sidewalk	0.74	1.3	0.61	0.64		
18	E	Hard to concentrate	1.75	1.6	0.62		0.57	
19	F	Walk around house in the dark	0.72	1.4	0.62			0.60
20	E	Afraid to stay home alone	0.55	1.3	0.51		0.65	
21	E	Feel handicapped	0.38	1.0	0.48		0.58	
22	E	Stressed relationship	0.53	1.2	0.53		0.68	
23	E	Depression	1.35	1.6	0.64		0.68	
24	F	Household responsibility	1.45	1.7	0.70			0.70
25	P	Bend over	1.75	1.6	0.65	0.73		

P: physical; E: emotional; F: functional.

**Table 4:** Results of the component analysis: five factors of Japan version and four factors of Chinese version—label (factor loading) of the corresponding items.

DHI	English version	Abbreviated	Taiwan 4 factor
8	Physical	Perform more ambitious activities	T1 (0.52)
11	Physical	Quick head movements	T1 (0.61)
25	Physical	Bend over	T1 (0.62)
14	Functional	Strenuous homework or yard work	T1 (0.48)
24	Functional	Job or household responsibilities	T1 (0.66)
18	Emotional	Hard to concentrate	T1 (0.61)
23	Emotional	Depressed	T1 (0.60)
16	Functional	Go for a walk by yourself	T2 (0.56)
19	Functional	Walk around house in the dark	T2 (0.58)
17	Physical	Walk down a sidewalk	T2 (0.44)
15	Emotional	Afraid people think you are intoxicated	T2 (0.47)
20	Emotional	Afraid to stay home alone	T2 (0.70)
9	Emotional	Afraid to leave home alone	T2 (0.56)
10	Emotional	Embarrassed in front of other	T2 (0.40)
21	Emotional	Feel handicapped	T2 (0.57)
22	Emotional	Stressed relationship with family/friends	T2 (0.63)
12	Functional	Avoid heights	T3 (0.51)
5	Functional	Get into or out of bed	T3 (0.46)
13	Physical	Turning over in bed	T3 (0.57)
4	Physical	Walk down the supermarket aisle	T3 (0.48)
1	Physical	Look up	T3 (0.54)
2	Emotional	Feel frustrated	T4 (0.50)
3	Functional	Restrict travel	T4 (0.66)
6	Functional	Restrict participation in social activities	T4 (0.59)
7	Functional	Hard to read	T4 (0.45)

**Table 5:** Spearman's correlation coefficients (*P* value) of questionnaires.

	BAI	BDI	ESS	PSQI
DHI-total	0.54 (<0.01)	0.46 (<0.01)	0.24 (<0.01)	0.38 (<0.01)
DHI-emotional	0.54 (<0.01)	0.50 (<0.01)	0.19 (<0.01)	0.37 (<0.01)
DHI-physical	0.48 (<0.01)	0.39 (<0.01)	0.26 (<0.01)	0.34 (<0.01)
DHI-function	0.49 (<0.01)	0.38 (<0.01)	0.21 (<0.01)	0.35 (<0.01)
T1	0.50 (<0.01)	0.43 (<0.01)	0.26 (<0.01)	0.36 (<0.01)
T2	0.49 (<0.01)	0.42 (<0.01)	0.17 (<0.01)	0.34 (<0.01)
T3	0.44 (<0.01)	0.34 (<0.01)	0.20 (<0.01)	0.32 (<0.01)
T4	0.42 (<0.01)	0.36 (<0.01)	0.18 (<0.01)	0.29 (<0.01)

**Table 6:** Result of a regression model with and without propensity score (PS).

	Without PS		With PS	
Outcome	Group effect	*R*-square	Group effect	*R*-square
Total score	17.62^∗^	0.13	6.79^∗^	0.32
DHI-function	6.14^∗^	0.09	1.71	0.26
DHI-physical	6.07^∗^	0.16	3.41^∗^	0.28
DHI-emotional	5.41^∗^	0.10	1.66	0.30
Factor T1	6.41^∗^	0.13	2.84^∗^	0.28
Factor T2	4.71^∗^	0.07	1.10	0.23
Factor T3	2.57^∗^	0.07	0.86	0.20
Factor T4	3.93^∗^	0.12	1.98^∗^	0.24

## Data Availability

The data used to support the findings of this study are available from the corresponding author upon request.
